The article "Pattern and In-Hospital Mortality of Thoracoabdominal Injuries Associated with Motor Vehicle Accident-Related Head Injury: a Single-Center Retrospective Study" was retracted in 2023. Reasons: signs of a paper mill; compromised peer review; unreliable results or conclusions.

# Pattern and In-Hospital Mortality of Thoracoabdominal Injuries Associated with Motor Vehicle Accident-Related Head Injury: a Single-Center Retrospective Study

**DOI:** 10.1155/2022/3602838

**Published:** 2022-06-21

**Authors:** Walid M. Abd El Maksoud, Mubarak Ali Algahtany

**Affiliations:** ^1^Division of General Surgery, Department of Surgery, College of Medicine, King Khalid University, Abha, Saudi Arabia; ^2^Division of Neurosurgery, Department of Surgery, College of Medicine, King Khalid University, Abha, Saudi Arabia

## Abstract

**Aim:**

To determine the pattern and in-hospital mortality of thoracoabdominal injuries associated with head injuries (HI) due to motor vehicle accidents. *Settings and Design.* A single-center retrospective study in a tertiary care hospital, level 1 trauma center in the southern region of Saudi Arabia.

**Methods and Materials:**

Descriptive analysis was conducted to evaluate sex, age, types of head injury, associated thoracoabdominal injuries, particular admission day, duration of hospital stay, and discharge category, and associations between different variables and outcomes were analyzed.

**Results:**

The cohort had a mean age of 26.9 ± 15.8 years, with a predominance of men (86.9%). Thoracoabdominal injuries were present in 6.8% of MVA-related HI, and 14.3% of victims expired during their hospital stay, mostly within the first 10 days. All expired patients had posttraumatic brain lesions. Moreover, there was a significant association between intensive care unit (ICU) admission and poor prognosis.

**Conclusions:**

Existence of posttraumatic brain lesions and requirement of ICU admission are significant variables affecting outcomes in patients with motor vehicle-associated HI with concomitant thoracoabdominal trauma in this study. Patients who survived the first 10 days after trauma seemed to have a better prognosis. More efforts are needed to reduce the health burden of this lethal injury.

## 1. Introduction

Traumatic head injury (HI) may cause damage to the scalp, skull, or brain. When the brain is affected, it is called traumatic brain injury (TBI) [1]. TBI, the “silent epidemic,” is a serious medical condition with the highest contribution to deaths and disabilities worldwide compared to any other traumatic insult [2]. TBI is associated with a mortality rate of 30 per 100,000 and an estimated 50,000 deaths in the United States annually [3]. Management of HI should target both the immediate impact of injury and its manifestation, and measures to prevent complications [4].

Motor vehicle accidents (MVAs) are the main causes of TBI in Saudi Arabia [5, 6]. Furthermore, MVAs are considered the main causes of TBI in developing countries [7, 8]. On the other hand, falls are considered the leading cause of TBI in North America and Europe [9, 10]. The effects of MVAs are usually variable, resulting in polytrauma. MVA outcomes may be affected by many factors, such as gender, age, type of collision, and speed of the vehicle [11, 12]. Traffic regulations and infrastructure may influence TBI incidence and outcomes in different regions of the world [2].

The article "Pattern and In-Hospital Mortality of Thoracoabdominal Injuries Associated with Motor Vehicle Accident-Related Head Injury: a Single-Center Retrospective Study" was retracted in 2023. Reasons: signs of a paper mill; compromised peer review; unreliable results or conclusions.

Head injuries lead to approximately 34% of all traumatic deaths, with an increased risk of mortality in older age groups [3, 13]. Thoracic and abdominal traumas are common among victims of MVAs [14, 15]. Thoracic injury is considered the second most common cause of mortality and major injury after HI [16]. Abdominal injury also contributes to trauma-related deaths following MVA and accounts for 10% of injuries due to MVAs [17].

Motor vehicle accidents resulting in polytrauma is usually managed in urgent circumstances. The apparent injury, especially if it is HI, may attract the most attention. This may affect the accurate diagnosis and proper management of hidden associated injuries [18, 19]. Extracranial injuries have been reported to significantly affect the outcome of patients with TBI when hospital admission is required [20]. Accordingly, knowledge of the pattern of associations between injuries helps predict outcomes. Furthermore, meticulous analysis of this association is of pivotal importance, especially after MVA, with its potential to cause multiorgan injuries [21]. However, very few prior studies have addressed the relationship between HI and associated thoracoabdominal injuries due to MVAs.

This study is aimed at determining the pattern and analyzing the in-hospital mortality of thoracoabdominal injuries associated with head injuries due to motor vehicle accidents.

## 2. Patients and Methods

This study had a retrospective design. Data for analysis were collected from the files of patients admitted to Aseer Central Hospital, the main tertiary hospital in Southern Saudi Arabia, from January 2010 to January 2020.

All patients aged 14 years or older, admitted due to MVA, and suffered from documented head injury in addition to thoracic and/or abdominal injuries were included in the study. Patients without associated thoracic or abdominal injuries and those with head injuries due to other causes were excluded from the study. Patients less than 14 years were treated in other hospital (Children's Hospital) according to the protocols of the Ministry of Health in Saudi Arabia.

The files of the patients were reviewed, and the following data set was recorded: demographic data, details of the head injuries and computed tomography (CT) reports if available, details of the thoracic and/or abdominal injuries, the need for critical care admission, duration of hospital stay, and prognosis on discharge.

The article "Pattern and In-Hospital Mortality of Thoracoabdominal Injuries Associated with Motor Vehicle Accident-Related Head Injury: a Single-Center Retrospective Study" was retracted in 2023. Reasons: signs of a paper mill; compromised peer review; unreliable results or conclusions.

### 2.1. Outcomes

The primary endpoints were as follows:

- Determination of the proportion of MVA-related HIs associated with thoracoabdominal injuries
- Determination of the pattern of thoracoabdominal injuries associated with MVA-related HI
- Determination of in-hospital outcomes of MVA-related HIs associated with thoracoabdominal injuries

The study was approved by the ethical committee of King Khalid University (ECM#2021-4001). All precautions were taken to conceal the identity of the patients.

### 2.2. Statistical Analysis

Statistical analysis of the data was performed using the Statistical Package for the Social Sciences “SPSS version 25 (SPSS, IBM, New York)”. Descriptive statistics were applied (i.e., frequency and percentage for categorical data, in addition to mean and standard deviation for quantitative data). The chi-square likelihood ratio was used to test the significance of the differences. Differences were considered statistically significant at *p* values less than 0.05.

## 3. Results

During the 10-year study period, 1,235 patients were admitted with MVA-related head injuries. Only 84 patients (6.8%) had associated thoracic and/or abdominal injuries. The patients included in our study had a mean age of 26.9 ± 15.8 years, and approximately half of the patients (52.4%) were between 20 and 40 years of age. Majority of our patients were male; the study population included 73 (86.9%) men and 11 (13.1%) women. Intra-axial lesions and head injuries with multiple intracranial lesions were the most common types of head injuries, occurring at 33.3% and 31.0%, respectively. The demographic and clinical data of the study group are shown in Table 1.

Regarding the type of thoracoabdominal injuries occurring with MVA-related HI, 58.3% of patients had associated chest injuries, of which lung contusion and pneumothorax constituted the most common thoracic injuries observed, at 19.0% and 13.1%, respectively (out of all studied patients). Abdominal injuries occurred in 38.1% of patients. Splenic injuries were the most common abdominal injuries (14.3%) (out of all studied patients). Only 3.6% of patients had both thoracic and abdominal injuries. Data regarding associated thoracic and abdominal injuries are presented in Table 2.

No specific variable was related to the type of head injury. Head injury combined with thoracoabdominal injuries is more common in older patients and in patients with other injuries. Associations between different variables and thoracoabdominal injuries, and the type of head injuries incurred are shown in Tables 3 and 4.

The article "Pattern and In-Hospital Mortality of Thoracoabdominal Injuries Associated with Motor Vehicle Accident-Related Head Injury: a Single-Center Retrospective Study" was retracted in 2023. Reasons: signs of a paper mill; compromised peer review; unreliable results or conclusions.

Studying the association between the different variables and the outcomes of our patients revealed that most deaths occurred within the first 10 days of injury. In addition, there is a significant association between intensive care unit (ICU) admission and poor prognosis. Associations between different variables and outcomes of head injury with thoracoabdominal injuries are shown in Table 5.

Multivariate binary logistic regression analysis (Table 6) revealed that patients' hospital stay and the need for admission to ICU were significantly associated with case fatality due to head injury (*p* = 0.017 and *p* < 0.001, respectively).

## 4. Discussion

According to reports by the World Health Organization, head trauma is responsible for hospitalization or death of 10 million people per year [22]. Although the total miles driven worldwide in 2020 was less than that in previous years due to the COVID-19 pandemic, 4.8 million roadway users were still seriously injured in MVAs, with an estimated 474 billion dollars cost to society. Approximately 1.3 million people died as a result of MVAs [23]. Motor vehicles are the main transportation methods in Saudi Arabia. The number of operating vehicles in Saudi Arabia in 2020 was estimated to be 10.03 million [24]. More than half a million MVAs occurred in Saudi Arabia in just one year, leading to 7,159 deaths and 40,000 injuries [25]. Accordingly, MVAs are considered to be the country's main cause of death, especially for 16- to 30-year-old males [26]. The accident-to-injury ratio in Saudi Arabia is very high, reaching up to 8 : 6, compared to the international ratio of 8 : 1 [25]. Detailed analysis may be required for a better understanding of this important health problem.

Head injury is considered a serious trauma due to the important and vital organs involved. MVAs are the leading causes of head injuries, especially TBI, with drastic consequences [27]. The faster the speed of the vehicle, the greater the magnitude of injuries and the incidence of associated deaths [28]. Head injuries, chest injuries, and abdominal hemorrhage are considered major causes of death in MVAs [17, 29]. Furthermore, a combination of abdominal, thoracic, and head injuries increases the risk of death [30].

Chest injuries represented approximately 60% of the associated injuries in our study, compared to approximately 40% for abdominal injuries. The most common thoracic injuries were lung contusions and pneumothorax. Chest injuries are common MVA-related injuries [17]. Mezue et al. [31] reported that the most common types of intrathoracic injuries are pneumothorax and hemothorax. However, their study did not exclusively include MVAs. Splenic injuries were the most commonly associated abdominal injuries in this study. The spleen is the most commonly injured viscus in blunt abdominal trauma [32].

The article "Pattern and In-Hospital Mortality of Thoracoabdominal Injuries Associated with Motor Vehicle Accident-Related Head Injury: a Single-Center Retrospective Study" was retracted in 2023. Reasons: signs of a paper mill; compromised peer review; unreliable results or conclusions.

In this study, no specific association was found between the type of head injury and the type of associated thoracoabdominal injury. Patients who suffered head injuries associated with thoracic and/or abdominal injuries were significantly found to suffer from other injuries, such as fractures and lacerations. This may be explained by the fact that the magnitude of the MVA can affect the extent and severity of injuries [28]. Head, thoracic, and abdominal injuries could be parts of multiple traumatic injuries in MVAs with a high magnitude rather than being connected with a specific pattern.

Chest and abdominal injuries are not merely associated with head injuries in MVAs, but could contribute to worsening of the outcome. Subsequent hypoxia or shock following chest or abdominal injuries may lead to secondary brain damage [33]. Early and accurate diagnosis and management of associated injuries can improve the survival of patients with severe head injuries [34]. Nevertheless, these associated injuries are usually overshadowed by an emphasis on head injury, which is the highest among other priorities.

The mortality rate of MVA-related HI associated with thoracoabdominal injuries in this study was 14.3%. This case fatality rate is comparable to the rates of death in MVA-related HI in other studies [35, 36]. The association between different variables and outcomes of MVA-related HI with thoracoabdominal injuries in this study revealed a significant association with ICU admission. All patients who died in our study had brain lesions. In addition, 9 out of the 12 deaths were in the first 10 days, which was found to be statistically significant. In general, head injuries may require a long hospital admission [37]. For patients suffering from MVA-related HI with thoracoabdominal injuries, the first 10 days seem to be crucial in determining their outcomes. Patients who survive the first 10 days had a better prognosis.

## 5. Limitations

This study was limited by its retrospective nature and by being a hospital-based study. It also lacked accident details and assessment of the severity of injury using validated scales, such as the injury severity score.

## 6. Conclusions

Existence of posttraumatic brain lesions and requirement of ICU admission are significant variables affecting outcomes in patients with motor vehicle-associated HI with concomitant thoracoabdominal trauma in this study. Patients who survived the first 10 days after trauma seemed to have a better prognosis. More efforts are needed to reduce the health burden of this lethal injury.

The article "Pattern and In-Hospital Mortality of Thoracoabdominal Injuries Associated with Motor Vehicle Accident-Related Head Injury: a Single-Center Retrospective Study" was retracted in 2023. Reasons: signs of a paper mill; compromised peer review; unreliable results or conclusions.

## Figures and Tables

**Table 1:** Demographics and outcome of motor vehicle accident-related traumatic head injuries associated with thoracoabdominal injuries (*n* = 84).

	No.	%
Age		
<20 years	29	34.5
20–40 years	44	52.4
>40 years	11	13.1
Mean ± SD	26.9 ± 15.8	
Gender		
Males	73	86.9
Females	11	13.1
Day of admission		
Weekday	64	76.2
Weekend	20	23.8
Diagnosis of head injury		
Extra-axial hematoma	15	17.9
Head injury, multiple lesions	26	31.0
Head injury, unspecified	3	3.6
Intra-axial lesion	28	33.3
Scalp injury	4	4.8
Skull fracture	8	9.5
Associated thoracoabdominal injuries		
Thoracic injuries	49	58.3
Abdominal injuries	32	38.1
Combined thoracoabdominal injuries	3	3.6
Hospital stay		
<10 days	28	33.3
10–20 days	16	19.0
>20 days	40	47.6
Discharge category		
Expired	12	14.3
Home	66	78.6
Transferred	6	7.1
Admission to ICU		
No	67	79.8
Yes	17	20.2
Other injuries		
No	49	58.3
Yes	35	41.7

**Table 2:** Associated thoracic and abdominal injuries.

Type of injury (*N* = 84)	No.	%
Thoracic injuries		
Thoracic injury, unspecified	8	9.5
Multiple chest injuries	4	4.8
Fracture ribs	5	6.0
Hemopneumothorax	1	1.2
Hemothorax	4	4.8
Pneumothorax	11	13.1
Lung contusion	16	19.0
Abdominal injuries		
Multiple abdominal injuries	1	1.2
Abdomen injury, unspecified	11	13.1
Pancreatic injury	1	1.2
Splenic injury	12	14.3
Hepatic injury	7	8.3
Combined thoracic and abdominal injuries		
Pneumothorax/liver injury	1	1.2
Lung contusion/spleen injury	1	1.2
Chest injury, unspecified/abdomen injury, unspecified	1	1.2

**Table 3:** Association between the different variables and thoracoabdominal injuries (*n* = 84).

Variables	Chest		Abdomen		Chest and abdomen		*p* value^†^
	No. (%)	AR	No. (%)	AR	No. (%)	AR	
Age							
<20 years	15 (51.7)	-0.9	13 (44.8)	0.9	1 (3.4)	0.0	**0.041**
20–40 years	27 (61.4)	0.6	17 (38.6)	0.1	0 (0.0)	-1.8	
>40 years	7 (63.6)	0.4	2 (18.2)	-1.5	2 (18.2)	2.8	
Gender							
Males	45 (61.6)	1.6	26 (35.6)	-1.2	2 (2.7)	-1.1	0.246
Females	4 (36.4)	-1.6	6 (54.5)	1.2	1 (9.1)	1.1	
Day of admission							
Weekday	37 (57.8)	-0.2	24 (37.5)	-0.2	3 (4.7)	1.0	0.434
Weekend	12 (60.0)	0.2	8 (40.0)	0.2	0 (0.0)	-1.0	
Hospital stay							
<10 days	19 (67.9)	1.3	9 (32.1)	-0.8	0 (0.0)	-1.2	0.235
10–20 days	9 (56.3)	-0.2	7 (43.8)	0.5	0 (0.0)	-0.9	
>20 days	21 (52.5)	-1.0	16 (40.0)	0.3	3 (7.5)	1.8	
Discharge condition							
Improved	36 (54.5)	-1.3	28 (42.4)	1.6	2 (3.0)	-0.5	0.264
Not improved	13 (72.2)	1.3	4 (22.2)	-1.6	1 (5.6)	0.5	
Discharge category							
Expired	9 (75.0)	1.3	3 (25.0)	-1.0	0 (0.0)	-0.7	0.284
Home	36 (54.5)	-1.3	28 (42.4)	1.6	2 (3.0)	-0.5	
Transferred	4 (66.7)	0.4	1 (16.7)	-1.1	1 (16.7)	1.8	
ICU admission							
No	38 (56.7)	**-0.6**	26 (38.8)	0.3	3 (4.5)	0.9	0.462
Yes	11 (64.7)	0.6	6 (35.3)	-0.3	0 (0.0)	-0.9	
Type of head injury							
Extra-axial hematoma	10 (66.7)	0.7	4 (26.7)	-1.0	1 (6.7)	0.7	0.247
Multiple lesions	16 (61.5)	0.4	8 (30.8)	-0.9	2 (7.7)	1.4	
Unspecified	2 (66.7)	0.3	1 (33.3)	-0.2	0 (0.0)	-0.3	
Intra-axial lesion	14 (50.0)	-1.1	14 (50.0)	1.6	0 (0.0)	-1.2	
Scalp injury	4 (100.0)	1.7	0 (0.0)	-1.6	0 (0.0)	-0.4	
Skull fracture	3 (37.5)	-1.3	5 (62.5)	1.5	0 (0.0)	-0.6	
Other injuries							
Yes	17 (48.6)	-1.5	15 (42.9)	0.8	3 (8.6)	2.1	**0.037**
No	32 (65.3)	1.5	17 (34.7)	-0.8	0 (0.0)	-2.1	

AR: adjusted residual. ^†^Based on the likelihood ratio chi-square statistic, *p* < 0.05 is significant.

The article "Pattern and In-Hospital Mortality of Thoracoabdominal Injuries Associated with Motor Vehicle Accident-Related Head Injury: a Single-Center Retrospective Study" was retracted in 2023. Reasons: signs of a paper mill; compromised peer review; unreliable results or conclusions.

**Table 4:** Association between the different variables and types of head injuries (*n* = 84).

Variables	Extra-axial hematoma		Multiple lesions		Unspecified		Intra-axial lesion		Scalp injury		Skull fracture		*p* value^†^
	No. (%)	AR	No. (%)	AR	No. (%)	AR	No. (%)	AR	No. (%)	AR	No. (%)	AR	
Age													
<20 years	4 (13.8)	-0.7	8 (27.6)	-0.5	2 (6.9)	1.2	9 (31.0)	-0.3	2 (6.9)	0.7	4 (13.8)	1.0	0.510
20–40 years	10 (22.7)	1.2	12 (27.3)	-0.8	1 (2.3)	-0.7	16 (36.4)	0.6	1 (2.3)	-1.1	4 (9.1)	-0.1	
>40 years	1 (9.1)	-0.8	6 (54.5)	1.8	0 (0.0)	-0.7	3 (27.3)	-0.5	1 (9.1)	0.7	0 (0.0)	-1.2	
Gender													
Males	15 (20.5)	1.7	23 (31.5)	0.3	2 (2.7)	-1.1	25 (34.2)	0.5	3 (4.1)	-0.7	5 (6.8)	-2.2	0.124
Females	0 (0.0)	-1.7	3 (27.3)	-0.3	1 (9.1)	1.1	3 (27.3)	-0.5	1 (9.1)	0.7	3 (27.3)	2.2	
Day of admission													
Weekday	13 (20.3)	1.1	16 (25.0)	-2.1	2 (3.1)	-0.4	22 (34.4)	0.4	4 (6.3)	1.1	7 (10.9)	0.8	0.233
Weekend	2 (10.0)	-1.1	10 (50.0)	2.1	1 (5.0)	0.4	6 (30.0)	-0.4	0 (0.0)	-1.1	1 (5.0)	-0.8	
Hospital stay													
<10 days	6 (21.4)	0.6	5 (17.9)	-1.8	0 (0.0)	-1.2	12 (42.9)	1.3	2 (7.1)	0.7	3 (10.7)	0.3	0.080
10–20 days	1 (6.3)	-1.3	4 (25.0)	-0.6	2 (12.5)	2.1	5 (31.3)	-0.2	2 (12.5)	1.6	2 (12.5)	0.5	
>20 days	8 (20.0)	0.5	17 (42.5)	2.2	1 (2.5)	-0.5	11 (27.5)	-1.1	0 (0.0)	-2.0	3 (7.5)	-0.8	
Discharge condition													
Improved	8 (12.1)	-2.6	22 (33.3)	0.9	2 (3.0)	-0.5	23 (34.8)	0.6	4 (6.1)	1.1	7 (10.6)	0.6	0.150
Not improved	7 (38.9)	2.6	4 (22.2)	-0.9	1 (5.6)	0.5	5 (27.8)	-0.6	0 (0.0)	-1.1	1 (5.6)	-0.6	
Discharge category													
Expired	4 (33.3)	1.5	4 (33.3)	0.2	0 (0.0)	-0.7	4 (33.3)	0.0	0 (0.0)	-0.8	0 (0.0)	-1.2	0.087
Home	8 (12.1)	-2.6	22 (33.3)	0.9	2 (3.0)	-0.5	23 (34.8)	0.6	4 (6.1)	1.1	7 (10.6)	0.6	
Transferred	3 (50.0)	2.1	0 (0.0)	-1.7	1 (16.7)	1.8	1 (16.7)	-0.9	0 (0.0)	-0.6	1 (16.7)	0.6	
ICU admission													
No	10 (14.9)	-1.4	21 (31.3)	0.2	2 (3.0)	-0.6	23 (34.3)	0.4	4 (6.0)	1.0	7 (10.4)	0.6	0.558
Yes	5 (29.4)	1.4	5 (29.4)	-0.2	1 (5.9)	0.6	5 (29.4)	-0.4	0 (0.0)	-1.0	1 (5.9)	-0.6	
Other injuries													
Yes	7 (20.0)	0.4	13 (37.1)	1.0	2 (5.7)	0.9	9 (25.7)	-1.3	0 (0.0)	-1.7	4 (11.4)	0.5	0.202
No	8 (16.3)	-0.4	13 (26.5)	-1.0	1 (2.0)	-0.9	19 (38.8)	1.3	4 (8.2)	1.7	4 (8.2)	-0.5	

AR: adjusted residual. ^†^Based on the likelihood ratio chi-square statistic, *p* < 0.05 is significant.

The article "Pattern and In-Hospital Mortality of Thoracoabdominal Injuries Associated with Motor Vehicle Accident-Related Head Injury: a Single-Center Retrospective Study" was retracted in 2023. Reasons: signs of a paper mill; compromised peer review; unreliable results or conclusions.

**Table 5:** Association between different variables and outcome of MVA-related HI with thoracoabdominal injuries (*n* = 84).

Variables	Expired		Home		Transferred		*p* value^†^
	No. (%)	AR	No. (%)	AR	No. (%)	AR	
Age							
<20 years	2 (6.9)	-1.4	24 (82.8)	0.7	3 (10.3)	0.8	0.438
20–40 years	7 (15.9)	0.4	35 (79.5)	0.2	2 (4.5)	-1.0	
>40 years	3 (27.3)	1.3	7 (63.6)	-1.3	1 (9.1)	0.3	
Gender							
Males	11 (15.1)	0.5	56 (76.7)	-1.1	6 (8.2)	1.0	0.335
Females	1 (9.1)	-0.5	10 (90.9)	1.1	0 (0.0)	-1.0	
Day of admission							
Weekday	8 (12.5)	-0.8	51 (79.7)	0.4	5 (7.8)	0.4	0.677
Weekend	4 (20.0)	0.8	15 (75.0)	-0.4	1 (5.0)	-0.4	
Hospital stay							
<10 days	9 (32.1)	3.3	19 (67.9)	-1.7	0 (0.0)	-1.8	**0.001**
10–20 days	1 (6.3)	-1.0	15 (93.8)	1.6	0 (0.0)	-1.2	
>20 days	2 (5.0)	-2.3	32 (80.0)	0.3	6 (15.0)	2.7	
ICU admission							
No	1 (1.5)	-6.7	64 (95.5)	7.5	2 (3.0)	-2.9	**<0.001**
Yes	11 (64.7)	6.7	2 (11.8)	-7.5	4 (23.5)	2.9	
Type of head injury							
Extra-axial hematoma	4 (26.7)	-2.8	8 (53.3)	-2.6	3 (20.0)	2.1	0.087
Multiple lesions	4 (15.4)	0.2	22 (84.6)	0.9	0 (0.0)	-1.7	
Unspecified	0 (0.0)	-0.7	2 (66.7)	-0.5	1 (33.3)	1.8	
Intra-axial lesion	4 (14.3)	0.0	23 (82.1)	0.6	1 (3.6)	-0.9	
Scalp injury	0 (0.0)	-0.8	4 (100.0)	1.1	0 (0.0)	-0.6	
Skull fracture	0 (0.0)	-1.2	7 (87.5)	0.6	1 (12.5)	0.6	
Site of associated injury							
Chest	9 (18.4)	1.3	36 (73.5)	-1.3	4 (8.2)	0.4	0.284
Abdomen	3 (9.4)	-1.0	28 (87.5)	1.6	1 (3.1)	-1.1	
Both	0 (0.0)	-0.7	2 (66.7)	-0.5	1 (33.3)	1.8	
Other injuries							
Yes	4 (11.4)	-0.6	28 (80.0)	0.3	3 (8.6)	0.4	0.765
No	8 (16.3)	0.6	38 (77.6)	-0.3	3 (6.1)	-0.4	

AR: adjusted residual. ^†^Based on the likelihood ratio chi-square statistic, *p* < 0.05 is significant.

**Table 6:** Binary logistic regression parameters for head injury patients' mortality.

Independent variables	*B*	S.E.	Wald	*p* value	Exp (*B*)	95% CI for Exp (*B*)	
						Lower	Upper
Age	-0.05	0.04	1.55	0.213	0.95	0.89	1.03
Site of injury	1.23	1.44	0.74	0.391	3.43	0.21	57.44
Hospital stay	1.75	0.74	5.65	**0.017** ^†^	5.78	1.36	24.53
Weekend	-0.01	1.393	0.00	0.995	0.99	0.07	15.20
Need for admission to ICU	5.90	1.619	13.26	**<0.001** ^†^	363.42	15.22	8675.37
Constant	-10.56	4.88	4.69	0.03	0.000		

^†^Statistically significant.

## Data Availability

Data will be available with the corresponding author to be sent on reasonable request.

The article "Pattern and In-Hospital Mortality of Thoracoabdominal Injuries Associated with Motor Vehicle Accident-Related Head Injury: a Single-Center Retrospective Study" was retracted in 2023. Reasons: signs of a paper mill; compromised peer review; unreliable results or conclusions.

## References

[1] Teasdale G. M. (1995). Head injury. *Journal of Neurology, Neurosurgery, and Psychiatry.*.

[2] Dewan M. C., Rattani A., Gupta S. (2019). Estimating the global incidence of traumatic brain injury. *Journal of Neurosurgery*.

[3] Kim A. H., Brooks M. R., Shaikh S. F. (2011). Traumatic Brain Injury. *Essential Clinical Anesthesia*.

[4] Rajajee V. (2019). Management of acute moderate and severe traumatic brain injury.

[5] Alghamdi F. S., Alsabbali D. M., Qadi Y. H., Albugami S. M., Lary A. (2021). Patterns and impact of traumatic brain injury at King Abdulaziz Medical City in Jeddah, Saudi Arabia: a retrospective cohort study. *Cureus*.

[6] Alnaami I., Alshehri S., Alghamdi S. (2019). Patterns, types, and outcomes of head injury in Aseer Region, Kingdom of Saudi Arabia. *Neuroscience Journal*.

[7] Bachani A. M., Koradia P., Herbert H. K. (2012). Road traffic injuries in Kenya: the health burden and risk factors in two districts. *Traffic Injury Prevention*.

[8] Seid M., Azazh A., Enquselassie F., Yisma E. (2015). Injury characteristics and outcome of road traffic accident among victims at Adult Emergency Department of Tikur Anbessa specialized hospital, Addis Ababa, Ethiopia: a prospective hospital based study. *BMC Emergency Medicine*.

[9] Peterson A. B., Kegler S. R. (2020). Deaths from fall-related traumatic brain injury—United States, 2008–2017. *Morbidity and Mortality Weekly Report*.

[10] Stranjalis G., Komaitis S., Kalyvas A. V. (2020). Recent trends (2010-2018) in traumatic brain injury in Greece: results on 2042 patients. *Injury*.

[11] Pawłowski W., Goniewicz K., Schwebel D. C., Shen J., Goniewicz M. (2019). Road traffic injuries in Poland: magnitude and risk factors. *European Journal of Trauma and Emergency Surgery*.

[12] Zhao X.-g., Wu J.-s., Zhao G.-f., Ma Y.-f., Zhang M., Gan J.-x., Xu S. W., Jiang G. Y. (2009). Risk factors for urban road traffic injuries in Hangzhou, China. *Archives of Orthopaedic and Trauma Surgery*.

[13] Viano D. C., Parenteau C. S., Xu L., Faul M. (2017). Head injuries (TBI) to adults and children in motor vehicle crashes. *Traffic Injury Prevention*.

[14] Brasel K. J., Nirula R. (2005). What mechanism justifies abdominal evaluation in motor vehicle crashes?. *Journal of Trauma and Acute Care Surgery*.

[15] Nirula R., Pintar F. A. (2008). Identification of vehicle components associated with severe thoracic injury in motor vehicle crashes: a CIREN and NASS analysis. *Accident Analysis & Prevention*.

[16] Schoell S. L., Weaver A. A., Talton J. W. (2018). Functional outcomes of motor vehicle crash thoracic injuries in pediatric and adult occupants. *Traffic Injury Prevention*.

The article "Pattern and In-Hospital Mortality of Thoracoabdominal Injuries Associated with Motor Vehicle Accident-Related Head Injury: a Single-Center Retrospective Study" was retracted in 2023. Reasons: signs of a paper mill; compromised peer review; unreliable results or conclusions.

[17] Arumugam S., Al-Hassani A., El-Menyar A. (2015). Frequency, causes and pattern of abdominal trauma: a 4-year descriptive analysis. *Journal of Emergencies, Trauma, and Shock*.

[18] Pfeifer R., Pape H.-C. (2008). Missed injuries in trauma patients: a literature review. *Patient Safety in Surgery*.

[19] Pfeifer R., Teuben M., Andruszkow H., Barkatali B. M., Pape H.-C. (2016). Mortality patterns in patients with multiple trauma: a systematic review of autopsy studies. *PLoS One*.

[20] Collaborators MCT (2008). Predicting outcome after traumatic brain injury: practical prognostic models based on large cohort of international patients. *BMJ*.

[21] Berkeveld E., Popal Z., Schober P., Zuidema W., Bloemers F., Giannakopoulos G. (2021). Prehospital time and mortality in polytrauma patients: a retrospective analysis. *BMC Emergency Medicine*.

[22] Hyder A. A., Wunderlich C. A., Puvanachandra P., Gururaj G., Kobusingye O. C. (2007). The impact of traumatic brain injuries: a global perspective. *Neuro Rehabilitation*.

[23] National Safety Council (2021). *Motor Vehicle Deaths in 2020 Estimated to Be Highest in 13 Years, Despite Dramatic Drops in Miles Driven*.

[24] Alkhathlan K. M., Alzahrani M. G., Aldosari K. H., Alsheddi M. I., Alqeair A. A. (2019). Traumatic spinal injuries in the Kingdom of Saudi Arabia: a study of associated injuries, management and mortality. *The Pan African Medical Journal*.

[25] Mansuri F. A., Al-Zalabani A. H., Zalat M. M., Qabshawi R. I. (2015). Road safety and road traffic accidents in Saudi Arabia: a systematic review of existing evidence. *Saudi Medical Journal*.

[26] WHOD, V (2009). *Global status report on road safety: time for action: World Health Organization*.

[27] Heegaard W., Biros M. (2007). Traumatic brain injury. *Emergency Medicine Clinics of North America*.

[28] Jurewicz C., Sobhani A., Woolley J., Dutschke J., Corben B. (2016). Exploration of vehicle impact speed - injury severity relationships for application in safer road design. *Transportation Research Procedia*.

[29] Luchter S., Smith A., Wang J. (1998). Fatal injuries in light vehicle crashes-time to death and cause of death. *Annual Proceedings/Association for the Advancement of Automotive Medicine*.

[30] Pimentel S. K., Sawczyn G. V., Mazepa M. M., Rosa F. G. G., Nars A., Collaço I. A. (2015). Risk factors for mortality in blunt abdominal trauma with surgical approach. *Revista do Colégio Brasileiro de Cirurgiões*.

[31] Mezue W. C., Ndubuisi C. A., Erechukwu U. A., Ohaegbulam S. C. (2012). Chest injuries associated with head injury. *Nigerian Journal of Surgery*.

[32] Shamim S. M., Razzak J. A., Umer S. M., Chawla T. (2011). Splenic injury after blunt abdominal trauma: an unusual presentation. *The Journal of Emergency Medicine*.

The article "Pattern and In-Hospital Mortality of Thoracoabdominal Injuries Associated with Motor Vehicle Accident-Related Head Injury: a Single-Center Retrospective Study" was retracted in 2023. Reasons: signs of a paper mill; compromised peer review; unreliable results or conclusions.

[33] Hellewell S. C., Yan E. B., Agyapomaa D. A., Bye N., Morganti-Kossmann M. C. (2010). Post-traumatic hypoxia exacerbates brain tissue damage: analysis of axonal injury and glial responses. *Journal of Neurotrauma*.

[34] Mohammad A., Branicki F., Abu-Zidan F. M. (2014). Educational and clinical impact of Advanced Trauma Life Support (ATLS) courses: a systematic review. *World Journal of Surgery*.

[35] Kiran Shankar H., Mohan Kumar K., Anand K. (2017). A clinical analysis of outcome in management of head injury in patients with highway road accidents. *International Journal of Research in Medical Sciences*.

[36] Urfi S. K., Amir A., Hoda M. F., Khalil S. (2013). Road traffic accidents with head injury: a study from western Uttar Pradesh. *Community Medicine*.

[37] Tardif P.-A., Moore L., Boutin A. (2017). Hospital length of stay following admission for traumatic brain injury in a Canadian integrated trauma system: a retrospective multicenter cohort study. *Injury*.

